# Alterations of Several Serum Parameters Are Associated with Preeclampsia and May Be Potential Markers for the Assessment of PE Severity

**DOI:** 10.1155/2020/7815214

**Published:** 2020-01-13

**Authors:** Zhongliang Duan, Cui Li, Wing Ting Leung, Jiangnan Wu, Mingyan Wang, Chunmei Ying, Ling Wang

**Affiliations:** ^1^Department of Clinical Laboratory, Hospital of Obstetrics and Gynecology, Fudan University, Shanghai, China; ^2^Laboratory for Reproductive Immunology, Hospital & Institute of Obstetrics and Gynecology, Shanghai Medical College, Fudan University, Shanghai, China; ^3^The Academy of Integrative Medicine, Fudan University, Shanghai, China; ^4^Shanghai Key Laboratory of Female Reproductive Endocrine-related Diseases, Shanghai, China; ^5^Department of Clinical Epidemiology, Hospital of Obstetrics and Gynecology, Fudan University, Shanghai, China

## Abstract

The precise pathophysiological mechanisms of preeclampsia (PE) and preventative strategies remain unknown. Laboratory markers which can help in identifying PE patients from pregnant women and assessing the severity of PE during pregnancy are worthy to be explored. In this study, a retrospective case-control study was designed to assess whether the serum levels of albumin (ALB), total protein (TP), prealbumin (PA), alkaline phosphatase (ALP), lactic dehydrogenase (LDH), D-dimer, fibrinogen (Fbg), platelet (PLT) count, mean platelet volume (MPV), and platelet distribution width (PDW) can help in assessing PE and evaluate its severity. 256 pregnant women were enrolled and classified into 3 groups: mild preeclampsia (mPE, *n* = 85), severe preeclampsia (sPE, *n* = 78), and healthy normotensive controls (control, *n* = 93). Our result showed that the serum levels of ALP, LDH, and D-dimer were significantly higher in mild or severe PE patients compared with the healthy controls (66 (52.5-76.5) vs. 168 (141.5-201.25) vs. 182.5 (120-191.5), 152 (139.75-166.25) vs. 183.5 (163.25-307) vs. 282 (215.25-306), 1.05 (0.65-1.57) vs. 3.05 (2.25-4.08) vs. 5.65 (2.29-7.71)), while ALB, TP, and PA are lower (38 (37-42) vs. 31.5 (25.5-34.5) vs. 28.5 (24-33), 65 (63-68.25) vs. 56.5 (52-61) vs. 51.5 (49-58), 219.14 ± 68.25 vs. 167.88 ± 52.21 vs. 143.22 ± 50.46). On the other hand, compared with the mPE group, the sPE group showed significantly lower PLT count but higher level of LDH, D-dimer, and Fbg. No significant differences in MPV or PDW were found between any of the two groups. In conclusion, the above markers except for the MPV and PDW may be correlated with PE severity in this patient cohort, indicating possible values of these potential biomarkers in auxiliary diagnosis and severity assessment of PE.

## 1. Introduction

Preeclampsia (PE) is a pregnancy-specific disease characterized by new-onset hypertension and proteinuria after 20 weeks of gestation associated with placental hypoperfusion. It is one of the major causes for fetal growth restriction, and in severe cases, it can progress into maternal multiorgan dysfunction or even mortality of both the mother and the newborn [1]. PE affects approximately 5–10% of pregnancies worldwide [2]. Pregnant women diagnosed with PE are often at a higher risk of future cardiovascular or cerebrovascular diseases [3]. The exact pathogenesis of PE remains controversial, while abnormal inflammation and immune responses [4, 5] and impaired coagulation-fibrinolysis systems [6, 7] are often mentioned. Among a number of possible causes of PE, the abnormal gestational trophoblast cell invasion and endothelial cell injuries are also widely studied. Deficient trophoblastic invasion into maternal myometrial spiral arteriole leads to the inadequate remodeling of the spiral arteries; the resulting abnormal implantation reduces the placental perfusion, thus causing the downstream hypoxia and maternal symptoms [8, 9]. The placental hypoperfusion may result in a state of hypoxia, yielding a state of excessive oxidative stress, angiogenic responses, and the release of antiangiogenic proteins and other inflammatory mediators which can lead to vascular endothelial damage and coagulation system activation [10]. The abnormal maternal metabolism can also adversely affect the intrauterine environment, aggravating the outcomes of PE [11]. Additionally, the roles of perturbation of the renin-aldosterone-angiotensin II axis, immune adaption, and genetic susceptibility are also being investigated by many studies [12–14].

Timely and accurate identification of the pregnant women who are at risk of developing PE is crucial as they require close prenatal monitoring and treatment to achieve better pregnancy outcomes. PE is typically diagnosed using clinical criteria which is based on nonspecific markers and clinical presentation. Currently, there is no screening or standard diagnostic test approved for clinical use [15]. Besides, PE may exist atypically, present individual difference, or resemble other conditions. Therefore, in recent years, attempts have been made to find specific and practical laboratory markers for PE prediction and assessment. Research has shown that the angiogenic pathway in early gestation is altered and excess angiogenic factors are released by the placenta into maternal blood. Maternal soluble endoglin (sEng) and soluble fms-like tyrosine kinase-1 (sFlt1) may be possible markers in early gestational age for prediction of PE [16–18]. There are also studies suggesting that MPV was significantly higher in preeclamptic women than in healthy pregnant women and thus may be a promising biomarker for the PE detection and follow-up [19]. Systemic immune inflammation indices such as neutrophil-lymphocyte ratio (NLR) and monocyte-lymphocyte ratio (MLR) are also reported to be effective in clinical assessment, disease severity evaluation, and prognosis evaluation of PE [20]. Changes of serum trace elements like Ca, Cu, and Mg are reported to be associated with PE, while serum ceruloplasmin [21] and soluble LIGHT [22] are reported to have predictive value in PE.

There have been controversies regarding the value of several hematological parameters (such as D-dimer, Fbg, PLT, MPV, and PDW) and biochemical tests (such as ALB, TP, PA, ALP, and LDH) in PE prediction or in the evaluation of PE severity. For example, the value of platelet count and platelet indices in PE is supported by several studies; however, there are also studies that found no significance [23–25]. The significance of ALB in assessing the onset and severity of preeclampsia is also controversial [26, 27].

Our study is aimed at providing further data and outcomes on these topics in Chinese population. We hypothesize that the altered levels of biological makers take part in clinical assessment, disease severity evaluation, and prognosis of PE during pregnancy. The primary aim of this study is to compare the ten serum parameters (ALB, TP, PA, ALP, LDH, D-dimer, Fbg, PLT, MPV, and PDW) of mild and severe preeclampsia patients at the time point they met diagnosis criteria with the normotensive controls, in order to investigate whether these parameters are correlated with PE or have a significant difference between sPE and mPE patients. Our study also hopes to provide further insight into the investigation of laboratory markers for PE clinical assessment and disease severity evaluation.

## 2. Methods

### 2.1. Patients and Controls

Data collection was approved by the Ethics Committee of the Obstetrics & Gynecology Hospital affiliated to Fudan University, and written informed consents were obtained from all cases. In this case-control retrospective study, a total of 256 pregnant women including 163 PE patients and 93 normotensive healthy controls were recruited from the obstetric outpatient clinic and inpatient department of the Obstetrics & Gynecology Hospital affiliated to Fudan University, during the time from June 2017 to June 2018. The recruitment of PE patients was consecutive. The enrolled controls were normal in blood pressure and immune system profile and were matched with the PE patients in gestational age and maternal prepregnancy body weight. Only pregnant women who have received all their antenatal examinations and delivered in our hospital were included in this study. PE is diagnosed according to the 2002 Practice Bulletin of American College of Obstetrics and Gynecology (ACOG) guidelines [28]. PE patients were further classified as mild preeclampsia (*n* = 85) and severe preeclampsia (*n* = 78). Preeclampsia is considered severe if systolic blood pressure (SBP) is ≥160 mm Hg or diastolic blood pressure (DBP) is ≥110 mm Hg or at least one of the following clinical symptoms occurred: renal insufficiency, pulmonary edema, microvascular disease, thrombocytopenia, impaired liver function, and peripheral severe organ involvement (visual impairment and headache) [29]. Patients were considered to have mild PE if they met the diagnostic criteria of preeclampsia but not the criteria for severe PE. Patients presented with other obstetric or systemic diseases were excluded from this study, which includes chronic hypertension, preexisting renal disease, immunological diseases, and multiple pregnancies HELLP syndrome. Pregnant women with other known medical complications which can affect the level of examined serum biomarkers, such as reproductive tract infections, recurrent spontaneous abortion, immunological diseases, and genetic diseases, were also excluded from this study.

### 2.2. Sample Collection and Analysis

Blood samples were collected as soon as the diagnosis of PE was confirmed and were tested within 2 hours. 2 mL of venous blood sample was collected into a test tube with EDTA-K-2 anticoagulant and was tested for whole blood count using Sysmex XN1000 hematology analyzer (Sysmex Corporation, Japan). Blood coagulative function was performed on a Sysmex CS5100 hematology analyzer (Sysmex Corporation, Japan) with another 2 mL of venous blood collected. 3 mL of venous blood sample was collected without anticoagulants for biochemical test and was tested by using Hitachi 7600 automatic analyzer (Hitachi Corporation, Japan). The above tests were conducted according to the manufacturer's instructions. The test results of serum ALB, TP, PA, ALP, LDH, D-dimer, Fbg, PLT, MPV, and PDW were all recorded. All these laboratory parameters were tested in our clinical laboratory, according to the ISO15189 standards.

### 2.3. Statistical Analysis Approach

The demographic and medical information of all enrolled pregnant women were obtained from medical records. The normality was analyzed by the Shapiro-Wilk test. The data of continuous variables were represented as *X* (mean) ± SD (standard deviation) or median and interquartile range. The categorical data were represented as percentage (%). Continuous data were compared within groups by the independent-samples *t*-test, one-way ANOVA, or Kruskal-Wallis test. The categorical data were analyzed by the chi-square test. Correlations between the parameters and the onset of PE were evaluated by the Pearson correlation coefficient (*r*). These biomarkers' values to evaluate PE were calculated by a receiver operating characteristic (ROC) curve. The area under curve (AUC) was calculated to evaluate the predictive powers. Each cutoff point was assessed by searching for the maximum Youden's index (sensitivity + specificity–1). SPSS 19.0 software was used for statistical analysis. *p* < 0.05 was considered statistically significant.

## 3. Results

### 3.1. Maternal Clinical and Demographic Characteristics Comparison between the mPE, sPE, and Control Groups

A total of 256 pregnant women were included in this study. Patients were divided into three groups: sPE (*n* = 78), mPE (*n* = 85), and healthy normotensive (control, *n* = 93) groups. Demographic and essential features of the three groups including age, gravidity, gestational age, vaginal delivery, and cesarean section rates are shown in Table 1. The average age of the sPE group patients is 32.22 ± 2.71, while the average age of the mPE group and healthy control group is 28.06 ± 2.84 and 29.38 ± 5.14 years, respectively. Compared to the control and mPE groups, women who developed sPE are higher in age (*p* < 0.05). There is no significant difference among the three groups with respect to gravidity (*p* > 0.05). Moreover, delivery time of the sPE group is significantly earlier than the control and mPE groups (*p* < 0.05). It is notable that compared with the control group, the sPE and mPE groups have higher rate of cesarean delivery, that is, lower rate of vaginal delivery (*p* < 0.001). There is a significant difference between the mPE and sPE groups regarding gestational age at delivery and delivery mode of vaginal or cesarean delivery.

### 3.2. Analysis of Biochemical Markers in the Three Groups

The levels of each tested serum parameter are shown in Table 2. The comparisons between the three groups are presented as *p* values demonstrated. As shown in Table 2, the ALB, TP, PA, ALP, LDH, and D-dimer levels of the control group are significantly different from those of the sPE and mPE groups. Specifically, the ALB, TP, and PA serum levels of the control group are higher than the sPE and mPE groups. On the contrary, for the ALP, LDH, and D-dimer, the control group is significantly lower. No significance is found by the comparison of ALB, TP, PA, and ALP levels between the mPE and sPE groups. The LDH and D-dimer of either the mPE or the sPE group are significantly higher than the control group, and the sPE group is higher than the mPE group. We also measured the serum level of Fbg, PLT, MPV, and PDW of the three groups. The result shows no significant difference between the control group and the mPE group in the levels of four parameters. However, by comparing the sPE patients with the healthy controls or mPE patients, the Fbg level is significantly higher and PLT is significantly lower in sPE patients. Significant difference of MPV level is found only between the control and sPE groups. There is no significant finding by comparing the PDW among the three groups.

### 3.3. Value of PE Evaluation by These Biomarkers

Correlation between these biomarkers and PE was evaluated by the Pearson correlation coefficient. The Pearson correlation coefficient and *p* values are shown in Table 3. The result suggests that PE is significantly positively correlated with biomarkers of ALP, LDH, and D-dimer and negatively correlated with ALB, TP, and PA.

The ROC curve is used to estimate the AUC of ALP, LDH, D-dimer, Fbg, MPV, and PDW which positively correlated with PE (Figure 1) and ALB, TP, PA, and PLT that negatively correlated with PE (Figure 2). The AUC in the prediction for PE of each marker is shown in Table 4.

## 4. Discussion

PE is a pregnancy complication characterized by new-onset hypertension and signs of abnormal metabolism or organ dysfunction. PE can lead to severe or even fatal complications for both the mother and the fetus. The pathogenesis of PE remains controversial.

In clinical practice, the laboratory index that can be obtained easily could help medical practitioners in monitoring PE directly. Thus, practical laboratory markers which can help in assessing the onset and severity of PE remain to be studied. In recent years, an increasing number of studies are giving attentions to the correlation between serum markers and severity of PE [30–32]. Soluble endoglin and soluble fms-like tyrosine kinase-1 [16], serum ceruloplasmin [21], and soluble LIGHT [22] in the early phrase of pregnancy are often reported to have possible value in PE prediction. However, so far, there is no reliable means. The onset of preeclampsia is considered a complicated pathophysiologic process associated with angiogenesis, hypoxia, oxidative stress, perturbation of the renin-aldosterone-angiotensin II axis, inflammation, immune maladaptation, and genetic susceptibility [15]. Thus, besides the definition of PE as the combination of high blood pressure and albuminuria in a pregnant woman, more clinical markers are needed for comprehensive assessment of PE.

In this retrospective study, we found more clinical markers that may be correlated with the onset and severity of PE, and they were easily measurable and available. We also found that the average age of the severe PE group was older than the other two groups, suggesting women that conceive at older age are at higher risk of developing PE. This is consistent with Sun et al.'s report [33]. Besides, we also found a significant difference in levels of ALB, TP, PA, ALP, LDH, and D-dimer between the healthy control group and either the mild or the severe PE group, suggesting that these biomarkers might have potential values in identifying PE patients from the pregnant women. PE often presents with proteinuria, which might lead to the low levels of ALB, TP, and PA in serum, and these markers may be useful for monitoring the progression of PE. The changes in the coagulation system and endothelial injury may lead to the abnormal expression of D-dimer, Fbg, and PLT in serum. The levels of LDH, D-dimer, Fbg, and PLT in the severe PE group were significantly different from the mild PE group, indicating potential value of auxiliary diagnosis in distinguishing mild and severe PE patients.

Platelet indices such as PLT, MPV, and PDW are widely available and cost-effective, facilitating its investigations in the prediction of PE [34, 35]. Freitas et al. [36] found that sPE patients had a significantly higher MPV. Dogan et al. [31] suggested that the increasing platelet turnover causes a decrease in the PLT, and an increase of MPV value and a decrease in PC/MPV ratio may play an important role in predicting the risk of PE. Our study showed similar results regarding the alterations of MPV and PLT in PE patients but different in the PDW level. The inconsistence in results may be due to the racial or methodological differences, which is worthy to be further studied. Consistent with previous studies [7, 37], D-dimer is significantly higher in PE patients, indicating a possible role of D-dimer in the pathology of PE.

The ROC curves and the Pearson correlation coefficient show significant positive correlation between PE and ALP, LDH, and D-dimer and negative correlation between PE and ALB, TP, and PA, which may be useful in daily clinical practice to predict the risk of PE.

Potential limitations of this study include that it is a single-center and retrospective study that still lacks evidence for use in clinical practice. Larger and multicenter prospective studies are still waited to be done to further verify the roles of the examined markers in assessment of PE severity and pregnancy outcomes.

In conclusion, the alterations of ALB, TP, PA, ALP, LDH, and D-dimer may have a role in the pathogenesis of PE or function in the development of PE. Our data suggest that these markers may have potential value in evaluating the risk and severity of PE. The serum parameters we studied can be readily derived and thus may be practical in daily clinical practice. Future large-scale prospective studies should further clarify the roles played by these parameters in the prediction of risk and severity of PE.

## Figures and Tables

**Figure 1:** ROC curve of each positively correlated biomarker. ROC curve was used to estimate each significantly positively correlated biomarker visually. The AUC of ALP, LDH, and D-dimer was more than 0.700. The AUC of Fbg, MPV, and PDW was less than 0.700.

**Figure 2:** ROC curve of each negatively correlated biomarker. ROC curve was used to estimate each significantly negatively correlated biomarker visually. The AUC of ALB, TP, and PA was more than 0.700. The AUC of PLT was less than 0.700.

**Table 1:** Summary of maternal characteristics of the control, mild preeclampsia, and severe preeclampsia groups.

	Control (*n* = 93)	mPE (*n* = 85)	sPE (*n* = 78)	*p* value
Age	29.38 ± 5.14	28.06 ± 2.84	32.22 ± 2.71∗	<0.05
Parity	1.14 ± 0.62	1.20 ± 0.68	1.06 ± 0.55	>0.05
Gestational age at sampling (weeks)	34.06 ± 4.62	33.12 ± 4.46	34.93 ± 4.13	>0.05
Gestational age at delivery (weeks)	39.04 ± 2.53	37.57 ± 3.44	35.69 ± 4.68^#^	<0.05
Highest SBP (mmHg)	118.22 ± 10.18∗∗	140.18 ± 18.34	155.41 ± 20.15	<0.01
Highest DBP (mmHg)	78.45 ± 11.29∗	94.35 ± 9.76	103.2 ± 10.18	<0.05
Renal function				
Blood urea nitrogen (mmol/L)	3.94 ± 1.16	4.13 ± 1.65	4.33 ± 1.58	>0.05
Uric acid (*μ*mol/L)	344.21 ± 57.17	405.91 ± 86.74	452.69 ± 93.33∗	<0.05
Creatinine (*μ*mol/L)	43.68 ± 10.23	48.38 ± 9.74	50.25 ± 9.66	>0.05
Urine albumin (g/24 h)	0.19 ± 0.12∗∗∗	1.92 ± 1.08	3.25 ± 1.12	<0.001
Vaginal delivery rate (%)	69∗∗∗	47	25	<0.001
Cesarean rate (%)	31∗∗∗	53	75	<0.001

Compared with the other two groups: ∗*p* < 0.05, ∗∗*p* < 0.01, ∗∗∗*p* < 0.001; compared with the control group: ^#^*p* < 0.05.

**Table 2:** Serum markers' values in different groups.

Marker	Control	mPE	sPE	Control vs. mPE	Control vs. sPE	mPE vs. sPE
ALB	38 (37-42)	31.5 (25.5-34.5)	28.5 (24-33)	<0.001	<0.001	0.2113
TP	65 (63-68.25)	56.5 (52-61)	51.5 (49-58)	0.0002	<0.001	0.4046
PA	219.14 ± 68.25	167.88 ± 52.21	143.22 ± 50.46	0.0002	<0.001	0.0555
ALP	66 (52.5-76.5)	168 (141.5-201.25)	182.5 (120-191.5)	0.0009	0.0001	0.4291
LDH	152 (139.75-166.25)	183.5 (163.25-307)	282 (215.25-306)	0.0022	<0.001	0.0444
D-dimer	1.05 (0.65-1.57)	3.05 (2.25-4.08)	5.65 (2.29-7.71)	<0.001	<0.001	0.0115
Fbg	3.58 ± 1.22	3.51 ± 1.15	4.12 ± 2.33	0.3969	0.0484	0.0470
PLT	232 (197-252.25)	211 (178-279)	169 (158-191.25)	0.4932	<0.001	0.0066
MPV	10.54 ± 2.03	10.69 ± 1.14	11.04 ± 2.51	0.2419	0.0137	0.1031
PDW	12.87 ± 3.54	13.5 ± 3.17	13.03 ± 4.26	0.1365	0.3810	0.2640

Data are presented as mean ± standard deviation (SD) when the parameters' distributions were normal distribution or median and interquartile ranges when skewed.

**Table 3:** Correlation between biomarkers and PE.

	ALB	TP	PA	ALP	LDH	D-dimer	Fbg	PLT	MPV	PDW
Pearson correlation coefficient	-0.770	-0.665	-0.622	0.560	0.571	0.628	0.183	-0.181	0.156	0.044
*p* value	0.000	0.000	0.000	0.000	0.000	0.000	0.092	0.096	0.152	0.686

**Table 4:** ROC curve of significant markers for evaluation of preeclampsia.

Variables	Cutoff value	Sensitivity	Specificity	AUC	Sig.	95% CI	
						Lower limit	Upper limit
ALB	34.000	100%	89.1%	0.954	<0.001	0.906	1.000
TP	59.500	97.5%	82.6%	0.939	<0.001	0.880	0.998
PA	184.500	95%	65.2%	0.882	<0.001	0.812	0.951
ALP	81.000	95.7%	77.5%	0.895	<0.001	0.822	0.968
LDH	183.500	73.9%	92.5%	0.899	<0.001	0.832	0.965
D-dimer	1.765	95.6%	85%	0.919	<0.001	0.858	0.980

## Data Availability

All my data in this manuscript were collected from patients of my hospital and approved by the Ethics Committee of the Obstetrics & Gynecology Hospital of Fudan University. All these data approved from my hospital can be provided for review process if needed.
